The article "Bioinformatics Analysis of Prognosis-Related Genes and Expression of CXCL8 in Colorectal Cancer" was published in 2022. Journal: Biomed Res Int.

# Bioinformatics Analysis of Prognosis-Related Genes and Expression of CXCL8 in Colorectal Cancer

**DOI:** 10.1155/2022/3149887

**Published:** 2022-07-06

**Authors:** Zhen Yao, Xue Pan, Wenyue Chen, Yongjian Pei, Chen Chen, Yongkang Huang, Songtao Liu, Yulong Liu

**Affiliations:** ^1^Department of Pulmonary and Critical Care Medicine, The Second Affiliated Hospital of Soochow University, Suzhou 215004, China; ^2^Department of Nuclear Accident Medical Emergency, The Second Affiliated Hospital of Soochow University, Suzhou 215004, China; ^3^Department of Ultrasound, The Second Affiliated Hospital of Soochow University, Suzhou 215004, China; ^4^State Key Laboratory of Radiation Medicine and Protection, School of Radiation Medicine and Protection, Collaborative Innovation Center of Radiological Medicine of Jiangsu Higher Education Institutions, Soochow University, Suzhou 215123, China

## Abstract

**Background:**

Colorectal cancer (CRC), one of the main causes of death, remains a leading cause of mortality in gastrointestinal cancer and tends to affect the younger generation. However, the pathological process of colorectal cancer is unclear. Exploring potential pathogenesis and therapeutic targets of CRC is significant as its high prevalence and high mortality. Nowadays, the rapid development of bioinformatics provides us an opportunity to explore potential molecular markers of CRC.

**Materials and Methods:**

First, three CRC gene chips with paracancerous controls were downloaded from the Gene Expression Omnibus (GEO) database. Second, after combining and batch correcting the three chips using the R language and Perl language, the differentially expressed genes (DEGs) were selected to investigate how they affect the CRC occurrence and development by GO and KEGG enrichment analysis. Third, based on the STRING website and the Cytoscape software, the protein-protein interaction (PPI) network was constructed and the core genes were screened out. Finally, through polymerase chain reaction (PCR) and immunohistochemistry (IHC), the expression and function of the core gene CXCL8 in CRC were explored.

**Results:**

GSE10950, GSE44076, and GSE75970, including 126 intestinal cancer samples and 126 paracancer samples, were screened as the datasets. 192 DEGs were screened, including 43 upregulated genes and 149 downregulated genes. Through the DEGs screened out, GO enrichment analysis, KEGG enrichment analysis, and the construction of PPI interaction network were carried out. Finally, according to the nodes and edges in the PPI network, the DEGs were sorted and the core genes were selected. Through basic experiments, the first ranked CXCL8 was further studied, and the results suggest that the expression of CXCL8 is related to the proliferation, migration, invasion, and even distant metastasis of CRC.

The article "Bioinformatics Analysis of Prognosis-Related Genes and Expression of CXCL8 in Colorectal Cancer" was published in 2022. Journal: Biomed Res Int.

**Conclusion:**

The present study showed that DEGs of CRC are associated with multiple tumor-related biological processes and signaling pathways. The core gene CXCL8 has the potential to be a new therapeutic target for CRC.

## 1. Introduction

Since the 21st century, the incidence and mortality of cancer are still growing rapidly worldwide. Bray et al. estimated in 2018 that 17 million new cancer cases and 9.5 million cancer deaths would occur worldwide [1]. CRC is universally acknowledged as the third most common tumor and the fourth most fatal tumor [2, 3]. Since the twenty-first century, Western pattern diet and lifestyle have had an increasing impact on human health, and the incidence rate of CRC has also increased [4, 5]. CRC includes colon cancer and rectal cancer, in which colorectal adenocarcinoma accounts for about 95% of all CRC. Risk factors for CRC include environment, family history, age, obesity, smoking, drinking, less exercise, and malnutrition [2, 6, 7]. The incidence rate of CRC is one of the common causes of cancer-related deaths, accounting for 10% of all new cancer cases worldwide [8]. In the treatment of CRC, early diagnosis is of great significance, so it is necessary to dig out more CRC biomarkers.

Nowadays, systemic chemotherapy is still the main method for the treatment of CRC. However, with the advent of targeted drugs such as anti-VEGF and anti-EGFR, the treatment of CRC has made a major breakthrough. In addition, new targets such as scaffold attachment factor B (SAFB) [9], centromeric protein H (cenph) [10], dematin actin binding protein (dmtn) [11], and rhombic structural protein 1 (rhbdd1) [12] have also been widely concerned and studied. With the rapid development of bioinformatics technology, plenty of clinical and genetic data are disclosed, which provides rich resources for basic and clinical research of tumors. Through various public databases, we can further study the pathogenesis of cancer and explore new tumor markers and potential therapeutic targets of CRC.

In this study, three gene chips including GSE10950 [13], GSE44076 [14], and GSE75970 [15] were screened from the geo database. The three gene chips that met the inclusion criteria were combined and batch corrected, and then, the DEGs in CRC and adjacent normal tissues were screened by R language and Perl language. GO enrichment analysis, KEGG enrichment analysis, and protein interaction network (PPI) construction were carried out according to the screened DEGs. Through GO and KEGG enrichment analyses, the role of DEGs in cell components, molecular functions, biological processes, various conduction pathways, and related biological pathways was further explored. According to the number of PPI nodes, the top 15 genes were screened, and the first row CXCL8 was selected for further analysis.

The article "Bioinformatics Analysis of Prognosis-Related Genes and Expression of CXCL8 in Colorectal Cancer" was published in 2022. Journal: Biomed Res Int.

Finally, the expression and function of CXCL8 in CRC were verified by polymerase chain reaction (PCR), and the correlation between the clinical characteristics and CXCL8 expression was analyzed by immunohistochemistry (IHC).

## 2. Materials and Methods

### 2.1. Microarray Data Information

The three gene chips used in this study were selected from the official website of geo (http://www.ncbi.NLM.NIH.Gov/GEO/). In order to reduce heterogeneity, the gene chips corresponding to CRC tissue and its adjacent normal tissue were selected. In addition, all data were downloaded from GPL platform, and all experimental methods were high-throughput sequencing. As shown in Table 1, these chips consisted of 126 colorectal cancer samples and 126 adjacent control samples, namely, GSE10950, GSE 44076, and GSE 75970. Sva package was used to eliminate the batch effects of these three datasets [16]. Through limma package and empirical Bayesian method [17], the DEGs were screened, and statistically significant DEGs were defined as *p* < 0.05 and |logFC| ≥ 2.

### 2.2. GO and KEGG Enrichment Analyses

In order to further research the role of DEGs in the occurrence and development of CRC, the GO and KEGG enrichment analyses were carried out through clusterProfiler package. A *p* value < 0.05 was regarded as a significant enrichment [18]. Through GO enrichment analysis, the molecular functions (MF), cellular components (CC), and biological processes (BP) involved in different genes were interpreted. KEGG enrichment analysis was conducted to explore the role of DEGs in various signal transduction pathways in the human body.

### 2.3. Integration of the PPI Network

The protein-protein interaction (PPI) network was constructed by online database STRING. Search by gene name or sequence number, and select Homo sapiens as the species. After removing free genes and selecting confidence (0.7), we constructed the final PPI network. Then, the Cytoscape software was applied to explore the internal relationship and interaction of the screened proteins. Through Perl language, the nodes in the PPI network were counted to rank the DEGs.

### 2.4. Survival Analysis

CRC data with clinical characteristics were downloaded from TCGA database, and then, they were extracted, decompressed, and merged through Perl language. The expression data of CXCL8 was extracted by biomanager and limma package. The survival curves were finally plotted by the survival package, in which CXCL8 was divided into high expression group and low expression group based on the median expression level.

The article "Bioinformatics Analysis of Prognosis-Related Genes and Expression of CXCL8 in Colorectal Cancer" was published in 2022. Journal: Biomed Res Int.

### 2.5. Cell Culture

All human CRC cell lines (SW480, HCT-8, HR8348, and HIEC) were provided by the cell bank of Chinese Academy of Science. All cell lines were cultured at 37°C with 5% CO_2_ and 85% relative humidity in DMEM medium (Gibco, Thermo Fisher Scientific, Waltham, MA, USA) supplemented with 10% FBS (Gibco, Thermo Fisher Scientific, Waltham, MA, USA).

### 2.6. Cell Transfection

To knock down the expression of CXCL8, three CXCL8-targeted siRNAs were synthesized through GenePharma. The sequences of the three siRNAs are listed in Table 2. The day before cell transfection, the cells were inoculated on 6-well plates and 2 ml cell culture medium containing FBS (Gibco, Thermo Fisher Scientific, Waltham, MA, USA) and antibiotics was added. The cells in exponential growth period were selected to make the cells converge to 70-90% in 24 hours. 20 pmol RNA was added to 50 *μ*l opti MEM serum-free medium and gently mixed. 50 *μ*l serum-free opti MEM was diluted, and 2 *μ*l transfection reagent was added and then carefully mixed and stood at room temperature for 5 min. The diluted DNA and the mixed reagent were gently mixed and placed at room temperature for 20 minutes to form a complex. Add the mixed 100 *μ*l compound reagent into the hole of the culture plate, and then, gently shake the culture plate. After 4-6 h, the complex was removed and the medium was replaced. The temperature of CO_2_ incubator was set to 37°C, and the cells were incubated for more than 24-48 hours.

### 2.7. Quantitative Real-Time PCR

Total RNA was extracted by TRIzol reagent (Invitrogen, Carlsbad, CA, USA) from cultured cells according to the instructions provided by manufacturer. Through PrimeScript™ RT kit with gDNA Eraser (TaKaRa, China), the total RNA was reverse-transcribed into cDNA. Furthermore, qRT-PCR was performed by CFX Connect Real-Time PCR System (Bio-Rad) and SYBR Select Master Mix for CFX (Invitrogen). The amplification conditions were as follows: 95°C for 30s and then 40 cycles of 95°C for 10s, primer temperature 56°C for 20s, and 72°C for 1 min. The CT value data in the reaction were collected by setting the corrected threshold, real-time fluorescence quantitative PCR and 2-△△Ct method. The qRT-PCR primer pairs are listed in Table 3.

### 2.8. Cell Counting Kit-8 Assay

To detect the growth and proliferation of cells, the CCK-8 kit (Yeasen Biotechnology, Shanghai, China) was applied. The cells were plated in 96-well plates (3000 cells/well). The culture plates were precultured in an incubator for a while (37°C, 5% CO_2_). CCK-8 was added into 96-well plates at 0 h, 24 h, 48 h, and 72 h after transfection and then cultured in incubator for 1 h. The absorbance of cells at OD450 nm was measured by multifunctional microplate reader, and the IC50 value was calculated by GraphPad software.

The article "Bioinformatics Analysis of Prognosis-Related Genes and Expression of CXCL8 in Colorectal Cancer" was published in 2022. Journal: Biomed Res Int.

### 2.9. Wound Healing Assay

Wound healing assay was conducted to measure cell repairability and migration. 10 *μ* tip was used to make a mark on the cell layer in the central growth area. In order to remove the cells that do not adhere to the tube wall (crossed cells), the cells were washed with sterile PBS for 3 times and then changed them to the culture medium with 1% FBS serum (Gibco, Thermo Fisher Scientific, Waltham, MA, USA). The cells were cultured in a 5% CO_2_ incubator at 37°C for 24 hours. The growth of cells and the width of scratches were observed using a microscope at the beginning of culture and 24 hours after culture.

### 2.10. Transwell Migration and Invasion Assays

To detect the migration and invasive ability of cells, the Transwell assay was performed by Transwell apparatus (Corning, NY, USA). The colorectal cancer cells were digested by trypsin and then washed with PBS. None serum medium-treated cells were added into the upper cavity (1 × 10^5 cells per well), and DMEM medium containing 10% fetal bovine serum was added into the lower cavity. Except for 50 *μ*l diluted Matrigel (BD Biosciences, Franklin lakes, NJ) in the upper chamber, other steps in the invasion test were the same as those from the migration test. The cells were fixed, stained, and counted at the specified time. Three parallel experiments were required. Trypsin, PBS, and serum-free medium were all purchased from Thermo Fisher Scientific (Shanghai, China).

### 2.11. Immunohistochemistry (IHC)

64 specimens of colorectal cancer and its adjacent normal tissues were collected in the Department of Pathology of the Second Affiliated Hospital of Suzhou University and were made into pathological chips. Following the classical immunohistochemical protocol, the protein expression of CXCL8 was evaluated by mouse monoclonal to CXCL8 (1 : 500, ab18672, Abcam) antibody and anti-mouse IgG for IP secondary antibody (ab131368, Abcam). In this study, the results were analyzed and summarized by the Mattern semiquantitative method. The scoring system is listed in Table 4, and the final score was calculated following the formula in Table 4.

## 3. Results

### 3.1. DEGs in CRC and the Enrichment Analysis of These Genes

In this study, we used three datasets for joint analysis, with a total sample size of 252, consisting of 126 colorectal cancer samples and 126 adjacent cancer samples. All samples were combined for batch correction. During the screening of DEGs, the cutoff value was set as |log2 (fold change)| ≥ 2 , and the adjusted *p* value was < 0.05. Finally, 192 DEGs were obtained, including 43 upregulated genes and 149 downregulated genes. According to the DEGs, we mapped the heat map (Figure 1(a)) and volcano map (Figure 1(b)). Heat map can measure the similarity of expression between samples or genes, and volcano map can vividly show the distribution of DEGs.

The article "Bioinformatics Analysis of Prognosis-Related Genes and Expression of CXCL8 in Colorectal Cancer" was published in 2022. Journal: Biomed Res Int.

GO enrichment analysis was used to further explore the role of DEGs in colorectal cancer. In the cell components, it is mainly enriched in the structural components of the extracellular matrix. Molecular functions are mainly concentrated in the activities of various proteins, such as carbonate dehydratase activity, receptor ligand activity, signal receptor activator activity, hormone activity, chloride ion transmembrane transporter activity, metallopeptidase activity, inorganic anion transmembrane transport activity, alcohol dehydrogenase [NAD (P) +] activity and oxidoreductase activity (ch-oh group acting on donor, nad or NADP as receptor), hydrolase activity, and phosphodiester hydrolase activity. Biological processes are mainly concentrated in heparin binding and glycosaminoglycan binding. Bar chart (Figure 2(a)) was drawn at the same time.

As a result of KEGG enrichment analysis, the DEGs mainly involved in nitrogen metabolism, PPAR signaling pathway, mineral absorption, bicarbonate recovery in proximal tubules, fat digestion and absorption, pancreatic secretion, bile secretion, retinol metabolism, and so on. Bar chart (Figure 2(b)) was also drawn.

### 3.2. PPI Network and Cluster Analysis

192 DEGs were inputted into the official website of string. After removing free genes and selecting reliability (0.7), the final PPI network was constructed (Figure 3(a)). In addition, the interaction between candidate proteins was analyzed by Cytoscape software. The nodes and relationships of the constructed PPI network are counted and sorted. As shown in Figure 3(b), the top 15 genes from high to low were listed, and the highest-ranked CXCL8 was selected for further analysis.

### 3.3. Survival Analysis

In the TCGA database, 93 samples with survival data were selected for prognostic analysis, and the survival curve was drawn (Figure 4). The calculated *p* value was 0.026. The results showed that the high expression of CXCL8 suggested the poor prognosis of colorectal cancer.

### 3.4. Interpretation of PCR Results

Bioinformatics studies manifested that the expression of CXCL8 in CRC cells was significantly higher than that in normal colorectal cells. In order to verify the above results, the expression of CXCL8 in normal intestinal epithelial cells and a variety of CRC cells (HCT-8, SW480, and hr8348) was detected. The results suggested that the expression of CXCL8 in a variety of CRC cells is significantly higher than that in normal intestinal epithelial cells. In addition, as shown in Figure 5(a), the expression of CXCL8 in SW480 is the most obvious. Therefore, SW480 was finally selected as a tool cell.

The article "Bioinformatics Analysis of Prognosis-Related Genes and Expression of CXCL8 in Colorectal Cancer" was published in 2022. Journal: Biomed Res Int.

After constructing CXCL8 primers, three different siRNA sequences (si-cxcl8-1, si-cxcl8-2, and si-cxcl8-3) were designed and synthesized to downregulate the expression of CXCL8 in SW480, and the interference efficiency was detected by QRT PCR. As shown in Figure 5(b), si-cxcl8-2 has the best interference effect and was selected as the interference sequence in the next research.

### 3.5. Interpretation of Cell Function Experiment

Si-cxcl8-2 was used to downregulate the expression of CXCL8 in SW480 cells, and then, the growth and proliferation of SW480 cells was detected by cell counting kit-8 assay. As shown in Figure 5(c), by comparing the Si NC group with the Si CXCL8 group, it is found that downregulating CXCL8 could inhibit the growth and proliferation of SW480 cells. In addition, as a result of wound healing assay, Transwell migration test, and Transwell invasion test, the downregulated CXCL8 would inhibit the migration and invasion of CRC cells (Figures 6–8).

### 3.6. Interpretation of IHC Results

The pathological specimens and clinical information of 64 patients with CRC were collected, including 42 patients with colon cancer and 22 patients with rectal cancer. The obtained pathological specimens were made into pathological chips. The specific distribution of pathological chips is shown in Table 5. Immunohistochemical results showed that (1) the staining results in normal colorectal samples adjacent to cancer were negative (Figure 9(a)). (2) Among 64 CRC samples, 50 were negative (Figure 9(b)), 13 were positive, and 1 was strongly positive. (3) In 64 CRC samples, the positive rate was 21.9%. (4) The staining sites in CRC centrally distributed in the nucleus and cytoplasm (Figures 9(c) and 9(d)).

According to the results of IHC and the clinical data of related patients, a highly significant association between the expression of CXCL8 and the N stage (*p* = 0.007) and intravascular tumor thrombus (*p* = 0.032) was observed. However, it is irrelevant to gender, age, location of onset 1 and 2, degree of differentiation, T stage, M stage, etc. This operation is completed by IBM SPSS statistics 22. It should be noted that since 19 rectal cancer samples and 3 transverse colon cancer samples cannot be subdivided into left and right colon, there are only 40 samples in this group. Specific information can be found in Table 6.

The article "Bioinformatics Analysis of Prognosis-Related Genes and Expression of CXCL8 in Colorectal Cancer" was published in 2022. Journal: Biomed Res Int.

## 4. Discussion

In recent years, with the rapid development of China's economy, people's living conditions have generally risen, and the diet structure has also changed. The incidence rate and mortality rate of CRC gradually increase. This disease has become one of the main digestive diseases that affect the life span of our people. Although the diagnosis and treatment of CRC have improved in recent years, more than 1 million people still suffer from CRC and more than 0.6 million patients die of CRC every year. Nearly a quarter of CRC patients have developed distal metastasis once diagnosed. Even surgical resection of lesions cannot guarantee the nonrecurrence of advanced CRC. The 5-year survival rate for CRC is still low if the tumor relapses or metastasizes again after surgery [19]. Gene therapy of CRC takes full advantage of widespread high-throughput gene detection methods and developed tumor molecular biology, so the systematic treatment of CRC is no longer limited to traditional surgery, radiotherapy, and chemotherapy. At present, in addition to VEGF monoclonal antibody and EGFR monoclonal antibody, there are still few targeted drugs widely used in clinical practice. Therefore, it is particularly important to find new CRC targets with diagnostic and therapeutic significance.

Through GO enrichment analysis, we found that the molecular functions of DEGs are mainly enriched in the activity regulation of various proteins, such as enzymes, ligands, receptors, and transporters, among which the activity of oxidoreductase has attracted more attention in recent years. Studies have shown that oxidoreductase containing WW domain can encode a tumor suppressor, often changed in carcinoma [20]. New evidence has confirmed that WWOX is associated with steroid metabolism, bone metabolism, HDL-C metabolism, and glucose metabolism. The WWOX gene crosses the fragile site fra16d, which is one of the most active common fragile sites, where not only chromosome translocation occurs in multiple myeloma but also homozygous and hemizygous deletion appears in carcinoma and carcinoma-derived cell lines [21, 22]. The loss of WWOX, which often occurs in tumors, damaging the correction mechanism of many protein syntheses, tends to cause metabolic changes and leads to the occurrence of tumors.

GO enrichment analysis suggests that the biological process of DEGs can be enriched in chemokine receptor binding. In the occurrence and development of CRC, chemokines are closely related to the changes of the tumor cell microenvironment and play an important regulatory role in the biological process of tumor cells and lymphocytes. Among the core genes we screened, CXCL8 and CXCL1 both belong to the chemokine family. CXCL8 and its receptor CXCR2 are the two most significant upregulated chemokines in CRC [23]. Their role in cancer has been fully proved in different kinds of cancer cells, such as prostate cancer, gastric cancer, and colorectal cancer. CRC cells can express and secrete CXCL8 by autocrine, which can promote angiogenesis and neutrophil infiltration in tumor tissues, so as to enhance tumor proliferation and survival. CXCL1 is a potent proinflammatory mediator in inflammatory diseases and infection. A great number of studies have indicated that its high expression is closely associated with the onset and progression of various tumors [24, 25]. CXCL1 is regulated in different kinds of tumors. Activated CXCL1 is significantly related to the growth, proliferation, tumor angiogenesis, and metastasis of CRC cells [26–28]. KEGG enrichment analysis manifested that the DEGs were mainly involved in nitrogen metabolism, PPAR signaling pathway, mineral absorption, bicarbonate recovery in proximal tubules, fat digestion and absorption, pancreatic secretion, bile secretion, retinol metabolism, and so on.

The article "Bioinformatics Analysis of Prognosis-Related Genes and Expression of CXCL8 in Colorectal Cancer" was published in 2022. Journal: Biomed Res Int.

Recently, the role of redox in tumor occurrence and therapy has received more and more attention. Through bioinformatics, we found that the role of DEGs in CRC is closely related to redox reactions. GO and KEGG enrichment analyses suggest that the occurrence and development of CRC are related to oxidoreductase activity and the PPAR signal pathway. Tumor cells produce energy through aerobic glycolysis, where NAD acts as an electron receptor. Therefore, NADPH plays a vital role in controlling the high level of reactive oxygen species in rapidly proliferating cancer cells. NAD depletion has an inhibitory influence on tumor cells because the production and utilization of glucose are cut off [29]. Peroxisome proliferator-activated receptor (PPAR) is a member of the nuclear receptor family, divided into three different subtypes: PPAR*α* (NR1C1), PPAR *β*/*δ* (NR1C2), and PPAR *γ* (NR1C3). The activation or overexpression of PPAR *β*/*δ*, the most commonly expressed subtypes, is associated with increased tumor growth, given by studies of various tumor samples and cancer cell lines [30]. In the process of tumor occurrence and development, PPAR *β*/*δ* participates in lots of biological processes like oxidative stress homeostasis, epithelial-mesenchymal transition, differentiation of tumor-associated macrophages, and angiogenesis [31].

In this study, a total of 15 core genes were screened, and the first ranked CXCL8 was selected for further research. PCR results indicated that the expression of CXCL8 in CRC cells was significantly higher than that in normal intestinal epithelial cells. Gene function experiment showed that CXCL8 could significantly promote the proliferation, migration, and invasion of CRC cells. Furthermore, several investigations have indicated that CXCL8 plays a vital role in the process of the Ras signaling pathway initiating angiogenesis, which can promote tumor angiogenesis by promoting the expression of VEGR or directly acting on vascular endothelial cells [32]. CXCL8 can still mediate angiogenesis in CRC when HIF-1*α* gene is knocked out, which indicates that the proangiogenesis process of CXCL8 can be carried out without VEGF expression [33]. In 2011, Varney found that after applying CXCL8 receptor CXCR2 antagonist to CRC-bearing nude mice, tumor angiogenesis was significantly inhibited, and liver metastasis of CRC was also significantly inhibited [34]. The above studies showed that CXCL8 plays an essential role in the angiogenesis of CRC. IHC results showed that the positive rate of CXCL8 in CRC (21.9%) was significantly higher than which in adjacent normal tissues (0.0%). We collected the pathological specimens and clinical data of 64 patients with CRC and analyzed the correlation between the expression of CXCL8 and the corresponding clinical data. The results revealed that the positive expression of CXCL8 was associated with the N stage and the formation of intravascular tumor thrombus. In recent years, many IHC experiments indicated that the expression of CXCL8 was related to the tumor size, depth of invasion, lymphatic metastasis, and stage of CRC patients. In conclusion, we believe that the expression of CXCL8 may be related to lymph node metastasis and distal metastasis in CRC patients, but its specific mechanism needs to be further studied.

The article "Bioinformatics Analysis of Prognosis-Related Genes and Expression of CXCL8 in Colorectal Cancer" was published in 2022. Journal: Biomed Res Int.

## 5. Conclusion

Through bioinformatics, it can be found that the DEGs of CRC are mainly involved in the composition of extracellular matrix structural components, the activity regulation of various proteins, and the combination of various cellular metabolites. The occurrence and development of CRC are relevant to lots of biological processes, among which the oxidative stress mediated by differentially expressed genes plays an extremely vital role. 15 core genes were found as potential molecular markers of CRC, and CXCL8 was chosen for further study. The results suggest that the level of CXCL8 expression is relevant to the proliferation, migration, invasion, angiogenesis, and even distal metastasis of CRC. Its high expression may promote the progress of CRC and be related to the poor prognosis of CRC patients. Therefore, CXCL8 and its receptor are expected to become new markers and therapeutic targets of CRC.

## Figures and Tables

**Figure 1:** (a) Heat map. (b) Volcano map.

**Figure 2:** (a) Bar chart of GO enrichment analysis. (b) Bar chart of KEGG enrichment analysis.

**Figure 3:** (a) Protein interaction network. (b) Rank of core genes.

**Figure 4:** Survival curve.

**Figure 5:** The expression and function of CXCL8 in colorectal cancer. (a) The expression of CXCL8 in various colorectal cancer cell lines (^∗^*p* < 0.05; ^∗∗^*p* < 0.01; ^∗∗∗^*p* < 0.001). (b) The expression of CXCL8 in colorectal cancer cells detected by QRT PCR (SW480) (^∗^*p* < 0.05; ^∗∗^*p* < 0.01; ^∗∗∗^*p* < 0.001). (c) Cell counting kit-8 assay (SW480) (^∗^*p* < 0.05; ^∗∗^*p* < 0.01; ^∗∗∗^*p* < 0.001).

**Figure 6:** Wound healing assay (SW480) (^∗^*p* < 0.05; ^∗∗^*p* < 0.01; ^∗∗∗^*p* < 0.001).

**Figure 7:** Transwell migration assays (SW480) (^∗^*p* < 0.05; ^∗∗^*p* < 0.01; ^∗∗∗^*p* < 0.001).

**Figure 8:** Transwell invasion assays (SW480) (^∗^*p* < 0.05; ^∗∗^*p* < 0.01; ^∗∗∗^*p* < 0.001).

**Figure 9:** Immunohistochemical results. (a) Negative result of CXCL8 in normal tissue adjacent to carcinoma. (b) Negative result of CXCL8 in CRC. (c) CXCL8 dyed in the nucleus. (d) CXCL8 dyed in nucleus and cytoplasm.

**Table 1:** Information on normalization of microarray data.

Dataset name	Platform	Type of experiment	CRC	Normal	Total
GSE10950	GPL6104	Expression profiling by array	24	24	48
GSE44076	GPL13667	Expression profiling by array	98	98	196
GSE75970	GPL14550	Expression profiling by array	4	4	8
Total			126	126	252

**Table 2:** Sequences of the three siRNAs.

siRNA	siRNA sequence information
si-CXCL8-1	AAAGCUUUACAAUAAUUUCUGUU GAAAUUAUUGUAAAGCUUUCUUU
si-CXCL8-2	AGUUCUUUGAUAAAUUUGGGGUU CCAAAUUUAUCAAAGAACUGAUU
si-CXCL8-3	AGCUUUACAAUAAUUUCUGUGUU CAGAAAUUAUUGUAAAGCUUUUU

**Table 3:** qRT-PCR primer pairs.

Name	Primer sequence information
GAPDH-F	GAAGGTGAAGGTCGGAGTC
GAPDH-R	GAAGATGGTGATGGGATTTC
CXCL8-F	TCTGCAGCTCTGTGTGAAGG
CXCL8-R	TGGGGTGGAAAGGTTTGGAG

**Table 4:** Scoring system of immunohistochemistry.

Mark	0	1	2	3	4
Dyeing intensity	Not stained	Light yellow	Medium brownish yellow	Strong brownish brown	
Staining range	<5.0%	5.0%~25.0%	26.0%~50.0%	51.0%~75.0%	>75.0%

Final score = staining intensity∗staining range (positive product ≥ 3 and negative product<3).

**Table 5:** Specific distribution of pathological chips.

1 T	11T	21 T	31 T	41 T	51 T	61 T	1 N	11 N	21 N	31 N	41 N	51 N
2 T	12 T	22 T	32 T	42 T	52 T	62 T	2 N	12 N	22 N	32 N	42 N	52 N
3 T	13 T	23 T	33 T	43 T	53 T	63 T	3 N	13 N	23 N	33 N	43 N	53 N
4 T	14 T	24 T	34 T	44 T	54 T	64 T	4 N	14 N	24 N	34 N	44 N	54 N
5 T	15 T	25 T	35 T	45 T	55 T		5 N	15 N	25 N	35 N	45 N	55 N
6 T	16 T	26 T	36 T	46 T	56 T	61 N	6 N	16 N	26 N	36 N	46 N	56 N
7 T	17 T	27 T	37 T	47 T	57 T	62 N	7 N	17 N	27 N	37 N	47 N	57 N
8 T	18 T	28 T	38 T	48 T	58 T	63 N	8 N	18 N	28 N	38 N	48 N	58 N
9 T	19 T	29 T	39 T	49 T	59 T	64 N	9 N	19 N	29 N	39 N	49 N	59 N
10 T	20 T	30 T	40 T	50 T	60 T		10 N	20 N	30 N	40 N	50 N	60 N

T: tumor tissue; N: normal tissue.

The article "Bioinformatics Analysis of Prognosis-Related Genes and Expression of CXCL8 in Colorectal Cancer" was published in 2022. Journal: Biomed Res Int.

**Table 6:** Relationship between CXCL8 expression and clinicopathological features of colorectal cancer.

Grouping	CXCL8 expression		*p* value
	—	+	
Gender (*n* = 64)			
Male	29 (74.4%)	10 (25.6%)	*p* = 0.548
Female	21 (84.0%)	4 (16.0%)	
Age (*n* = 64)			
≤66	23 (71.9%)	9 (28.1%)	*p* = 0.226
>66	27 (84.4%)	5 (15.6%)	
Location 1 (*n* = 64)			
Colon	31 (73.8%)	11 (26.2%)	*p* = 0.403
Rectum	19 (86.4%)	3 (13.6%)	
Location 2 (*n* = 40)			
Left colon	13 (68.4%)	6 (31.6%)	*p* = 0.583
Right colon	16 (76.2%)	5 (23.8%)	
Differentiation (*n* = 64)			
High	3 (100.0%)	0 (0.0%)	*p* = 0.653
Moderate	43 (78.2%)	12 (21.8%)	
Low	4 (66.7%)	2 (33.3%)	
T stage (*n* = 64)			
T2	6 (100.0%)	0 (0.0%)	*p* = 0.317
T3	26 (72.2%)	10 (27.8%)	
T4	18 (81.8%)	4 (18.2%)	
N stage (*n* = 64)			
No metastasis	30 (93.8%)	2 (6.3%)	*p* = 0.007^∗^
Metastasis	20 (62.5%)	12 (37.5%)	
M stage (*n* = 64)			
No metastasis	43 (79.6%)	11 (204%)	*p* = 0.794
Metastasis	7 (70.0%)	3 (30.0%)	
Intravascular tumor thrombus (*n* = 64)			
No	42 (84.0%)	8 (16.0%)	*p* = 0.032^∗^
Yes	8 (51.7%)	6 (42.9%)	
AJCC stage (*n* = 64)			
I	4 (100.0%)	0 (0.0%)	*p* = 0.148
II	24 (88.9%)	3 (11.1%)	
III	15 (65.2%)	8 (34.8%)	
IV	7 (70.0%)	3 (30.0%)	

## Data Availability

All data included in this study are available from the corresponding author upon request.

## References

[1] Bray F., Ferlay J., Soerjomataram I., Siegel R. L., Torre L. A., Jemal A. (2018). Global cancer statistics 2018: GLOBOCAN estimates of incidence and mortality worldwide for 36 cancers in 185 countries. *CA: a Cancer Journal for Clinicians*.

[2] Dekker E., Tanis P. J., Vleugels J. L. A., Kasi P. M., Wallace M. B. (2019). Colorectal cancer. *The Lancet*.

[3] Schreuders E. H., Ruco A., Rabeneck L. (2015). Colorectal cancer screening: a global overview of existing programmes. *Gut*.

[4] Brody H. (2015). Colorectal cancer. *Nature*.

[5] Keum N., Giovannucci E. (2019). Global burden of colorectal cancer: emerging trends, risk factors and prevention strategies. *Nature Reviews Gastroenterology & Hepatology*.

[6] Buccafusca G., Proserpio I., Tralongo A. C., Rametta Giuliano S., Tralongo P. (2019). Early colorectal cancer: diagnosis, treatment and survivorship care. *Critical Reviews in Oncology/Hematology*.

[7] Thanikachalam K., Khan G. (2019). Colorectal cancer and nutrition. *Nutrients*.

The article "Bioinformatics Analysis of Prognosis-Related Genes and Expression of CXCL8 in Colorectal Cancer" was published in 2022. Journal: Biomed Res Int.

[8] Wong S. H., Yu J. (2019). Gut microbiota in colorectal cancer: mechanisms of action and clinical applications. *Nature Reviews Gastroenterology & Hepatology*.

[9] Jiao H. L., Ye Y. P., Yang R. W. (2017). Downregulation of SAFB sustains the NF-*κ*B pathway by targeting TAK1 during the progression of colorectal cancer. *Clinical Cancer Research*.

[10] Wu W., Wu F., Wang Z. (2017). CENPH inhibits rapamycin sensitivity by regulating GOLPH3-dependent mTOR signaling pathway in colorectal cancer. *Journal of Cancer*.

[11] Ye Y. P., Jiao H. L., Wang S. Y. (2018). Hypermethylation of DMTN promotes the metastasis of colorectal cancer cells by regulating the actin cytoskeleton through Rac1 signaling activation. *Journal of Experimental & Clinical Cancer Research*.

[12] Zhang M., Miao F., Huang R. (2018). RHBDD1 promotes colorectal cancer metastasis through the Wnt signaling pathway and its downstream target ZEB1. *Journal of Experimental & Clinical Cancer Research*.

[13] Jiang X., Tan J., Li J. (2008). DACT3 is an epigenetic regulator of Wnt/*β*-catenin signaling in colorectal cancer and is a therapeutic target of histone modifications. *Cancer Cell*.

[14] Solé X., Crous-Bou M., Cordero D. (2014). Discovery and validation of new potential biomarkers for early detection of colon cancer. *PLoS One*.

[15] Huang F. T., Chen W. Y., Gu Z. Q. (2017). The novel long intergenic noncoding RNA *UCC* promotes colorectal cancer progression by sponging miR-143. *Cell Death & Disease*.

[16] Leek J. T., Johnson W. E., Parker H. S., Jaffe A. E., Storey J. D. (2012). The sva package for removing batch effects and other unwanted variation in high-throughput experiments. *Bioinformatics*.

[17] Ried K., Finnis M., Hobson L. (2000). Common chromosomal fragile site FRA16D sequence: identification of the FOR gene spanning FRA16D and homozygous deletions and translocation breakpoints in cancer cells. *Human Molecular Genetics*.

[18] Paige A. J., Taylor K. J., Taylor C. (2001). WWOX: a candidate tumor suppressor gene involved in multiple tumor types. *Proceedings of the National Academy of Sciences of the United States of America*.

[19] Sparmann A., Bar-Sagi D. (2004). Ras-induced interleukin-8 expression plays a critical role in tumor growth and angiogenesis. *Cancer Cell*.

[20] Mizukami Y., Jo W. S., Duerr E. M. (2005). Induction of interleukin-8 preserves the angiogenic response in HIF-1*α*-deficient colon cancer cells. *Nature Medicine*.

[21] Varney M. L., Singh S., Li A., Mayer-Ezell R., Bond R., Singh R. K. (2011). Small molecule antagonists for CXCR2 and CXCR1 inhibit human colon cancer liver metastases. *Cancer Letters*.

[22] Verbeke H., Struyf S., Laureys G., Van Damme J. (2011). The expression and role of CXC chemokines in colorectal cancer. *Cytokine & Growth Factor Reviews*.

The article "Bioinformatics Analysis of Prognosis-Related Genes and Expression of CXCL8 in Colorectal Cancer" was published in 2022. Journal: Biomed Res Int.

[23] Yu G., Wang L. G., Han Y., He Q. Y. (2012). clusterProfiler: an R package for comparing biological themes among gene clusters. *OMICS: a Journal of Integrative Biology*.

[24] Abu-Remaileh M., Aqeilan R. I. (2015). The tumor suppressor WW domain-containing oxidoreductase modulates cell metabolism. *Experimental Biology and Medicine*.

[25] Ritchie M. E., Phipson B., Wu D. (2015). limma powers differential expression analyses for RNA-sequencing and microarray studies. *Nucleic Acids Research*.

[26] Pavlova N. N., Thompson C. B. (2016). The emerging hallmarks of cancer metabolism. *Cell Metabolism*.

[27] Planagumà A., Domènech T., Pont M. (2015). Combined anti CXC receptors 1 and 2 therapy is a promising anti-inflammatory treatment for respiratory diseases by reducing neutrophil migration and activation. *Pulmonary Pharmacology & Therapeutics*.

[28] Poutahidis T., Erdman S. E. (2016). Commensal bacteria modulate the tumor microenvironment. *Cancer Letters*.

[29] Wang Y., Liu J., Jiang Q. (2017). Human adipose-derived mesenchymal stem cell-secreted CXCL1 and CXCL8 facilitate breast tumor growth by promoting angiogenesis. *Stem Cells*.

[30] Han S., Zong S., Shi Q. (2017). Is Ep-CAM expression a diagnostic and prognostic biomarker for colorectal cancer? A Systematic Meta-Analysis. *EBioMedicine*.

[31] Kasashima H., Yashiro M., Nakamae H. (2017). Clinicopathologic significance of the CXCL1-CXCR2 axis in the tumor microenvironment of gastric carcinoma. *PLoS One*.

[32] Divella R., Daniele A., De Luca R. (2017). Circulating levels of VEGF and CXCL1 are predictive of metastatic organotropismin in patients with colorectal cancer. *Anticancer Research*.

[33] Cheng H. S., Tan W. R., Low Z. S., Marvalim C., Lee J. Y. H., Tan N. S. (2019). Exploration and development of PPAR modulators in health and disease: an update of clinical evidence. *International Journal of Molecular Sciences*.

[34] Wagner N., Wagner K. D. (2020). PPAR beta/delta and the hallmarks of cancer. *Cell*.

